The article "A Blockchain Framework to Secure Personal Health Record (PHR) in IBM Cloud-Based Data Lake" was published in 2022. Journal: Comput Intell Neurosci.

# A Blockchain Framework to Secure Personal Health Record (PHR) in IBM Cloud-Based Data Lake

**DOI:** 10.1155/2022/3045107

**Published:** 2022-04-12

**Authors:** Arvind Panwar, Vishal Bhatnagar, Manju Khari, Ahmad Waleed Salehi, Gaurav Gupta

**Affiliations:** ^1^University School of Information Communication and Technology, Guru Gobind Singh Indraprastha University, Delhi, India; ^2^Netaji Subhas University of Technology (East Campus), Geeta Colony, Delhi, India; ^3^Jawaharlal Nehru University, Delhi, India; ^4^Rana University, Kabul, Afghanistan. Yogananda School of Artificial Intelligence, Computers and Data Science, Shoolini University, Solan 173229, Himachal Pradesh, India; ^5^Yogananda School of Artificial Intelligence, Computers and Data Science, Shoolini University, Solan 173229, Himachal Pradesh, India

## Abstract

The health system in today's real world is significant but difficult and overcrowded. These hurdles can be diminished using improved health record management and blockchain technology. These technologies can handle medical data to provide security by monitoring and maintaining patient records. The processing of medical data and patient records is essential to analyze the earlier prescribed medicines and to understand the severity of diseases. Blockchain technology can improve the security, performance, and transparency of sharing the medical records of the current healthcare system. This paper proposed a novel framework for personal health record (PHR) management using IBM cloud data lake and blockchain platform for an effective healthcare management process. The problem in the blockchain-based healthcare management system can be minimized with the utilization of the proposed technique. Significantly, the traditional blockchain system usually decreases the latency. Therefore, the proposed technique focuses on improving latency and throughput. The result of the proposed system is calculated based on various matrices, such as F1 Score, Recall, and Confusion matrices. Therefore, the proposed work scored high accuracy and provided better results than existing techniques.

## 1. Introduction

IoT technologies lead the modern world into tremendous technological growth in terms of data management, communication, and information sharing [1]. With these developments, the modern world has gained massive advantages by utilizing technological equipment especially Bluetooth devices, WSN technology, Wi-Fi, Li-Fi, and RFID. Therefore, these smart devices help to simplify the difficulties in the communication of various fields, including education, agriculture, and transportation [2, 3]. Nowadays, these smart devices which are highly based on IoT, Artificial Intelligence (AI), Machine Learning, Virtual Reality (VR), and Augmented Reality (AR) are utilized everywhere [4, 5]. Moreover, the usages of smart technologies are inevitable in the medical domain due to their considerable advantages in maintaining patient records as well as providing effective treatment with advanced technological equipment. Also, the smart healthcare system has fetched the attention of many researchers to facilitate efficiency in the healthcare system. On the other hand, stakeholders are ready to invest and show their contribution to the healthcare system.

The most considerable factor of a smart health care system is faster identification and prediction of diseases automatically [6]. Here, healthcare-based smart technologies are discussed in detail utilizing the investigation of the development of smart technologies, and we also focused on its essential requirements for implementing a security system in the healthcare sector. The healthcare system is incorporated with a network-based electronic health management process along with the clinical imaging process. Therefore, the clinical records can be obtained as more effective in terms of security, accuracy, and time-sensitive patient data. By utilizing blockchain technology, the healthcare system is more enhanced with transparency and communication among patients and the practitioner. Various blockchain systems have been proposed in medical record management. However, more work is needed to better organize, understand, and evaluate the use of blockchain technology in the healthcare sector. However, the efficiency and effectiveness of the healthcare system will further inform, understand, and evaluate the application of blockchain technology to healthcare.

In the healthcare domain, privacy and security is a serious concern for maintaining patient confidential data [7]. The demand for a highly secured system is growing every day due to the individual need to disclose as per their requirements. To improve the security and privacy of healthcare data, tremendous secured systems are developed, especially HIPAA (Health Insurance Portability and Accountability Act of 1996), COBIT (Control Objectives for Information and Related Technologies), and DISHA (Digital Information Security in Healthcare Act). These are utilized to preserve patients' data in terms of maintaining the confidentiality of clinical data. In the medical field, privacy information should be handled by the healthcare providers where modification and deletion are controlled by them. Also, healthcare providers should give more concerns in terms of preventing unauthorized access by intruders. Because of the dramatic growth of healthcare data, enabling highly secured systems is essential. This is the reason why many countries including the USA have initiated the security standard and managed the data in terms of security analysis towards healthcare data.

Now the modern world is considered as a fourth generation of the healthcare industry where smart technologies are omnipresent in every medical field [8]. These technologies are highly required for managing and predicting diseases of patients, and the patient records are handled securely especially when executing the medical data transmission process. To maintain patient healthcare data, an Electronic Health Record (EHR) system is utilized by the healthcare provider. Moreover, the utilization of the EHR system is playing a vital role in healthcare data processing and maintaining. Therefore, the more considerable factors of healthcare records are free from threats and security issues. In case the system may not fulfill these requirements, the utilized system is not effective as a privacy requirement, and it is not suitable for obtaining the demand for security concerns.

The efficiency of the security system is highly based on maintaining its integrity based on avoiding duplicated and mismatched identifiers [9]. Moreover, the integrity of the system may get damaged due to security breaches and malicious activity. The attackers or hackers may access the particular patient's data by penetrating through the system if it is not having an appropriate security system [10]. This may lead to unauthorized access, data loss, and personal information being disclosed to the market without the appropriate permission from the concerned person [11]. Confidential data of patients consist of their contact numbers, addresses, names, medical details, etc. Because of this reason, patient data are confidential and an effective healthcare system is considered based on its security and privacy management mechanism [12]. By considering these challenges, an effective healthcare system is focused to be developed by many countries in terms of preventing cyber threats and maintaining confidentiality [13, 14]. These days, two-way communication-based architectures are being utilized in most healthcare systems, where the client and the server act as the sender and receiver of the system. However, the possibility of security is still high due to its open access; this causes the reason for the cyber intruders to access the specific data of the user.

Blockchain technology has nowadays fetched the attention of many researchers. It is mainly due to the dramatically enhanced cryptocurrencies, especially Bitcoin and Ethereum [15]. With the help of blockchain, the data can be stored and managed in a decentralized network; it is based on a trusted and fixed manner. The transparent nature of blockchain enables the complex strategy to deal with a ledger-based transaction via a network. It is connected with different computer controls from different components in the blockchain network. Moreover, this technique is highly focused to deal with speed calculation. This technique is incorporated with consensus protocol, the cryptography technique based on hash, the static ledger model, decentralized P2P networking, and data mining processes. All these processes are briefly discussed in the following section (Figures 1 and 2).

1. Consensus protocol: this level mainly deals with the service agreement between the client and the server; every transaction can be updated based on norms and conditions determined in the transaction. Moreover, this is the essential step/process in the blockchain network.
2. Cryptography: this is an essential step for enabling a security system to every field; therefore, the blockchain system utilized the SHA256 hash for preventing every transaction from data leakage. With the utilization of hash cryptography, the system has some considerable advantages, such as one-way cryptography, computation is faster and effective, and the collision can be avoided.
3. Static ledger: in a blockchain system, every transaction is noted and stored for effective data management processes. However, these records are not involved in the modification and editing process because it is static in nature.
4. Centralized P2P network: because of the complex and centralized nature of the system, every transaction has distributed nature in the network where various users are involved in updating or deleting their data.
5. Mining: in this network, blocks of nonce values are being utilized by miners for obtaining the hash values. Therefore, this system requires highly computational speed in order to get the reward. The considerable factor of the blockchain network is enabling the duplicate network to different places. The system can enable without any changes in the facility or healthcare provision network, within a particular region or throughout the world [16]. With this facility, the researchers, partners, and other parties can facilitate sharing healthcare records. For instance, the insurance service provider can enable their service to reach all over its consumers. Moreover, because of the distributed nature of blockchain enabled within the particular network, the communication is becoming simple; however, it must be checked whether the data within the network are correct, integrated, and consistent [17]. With this facility, the blockchain from one location can be distributed to many locations without changing its actual nature within the same location. Therefore, the new location can be determined within the network. Finally, these data are shared with the remaining network, and based on the latest data, accessing the latest data is possible.
6. Blockchain transaction processes: the blockchain process can be executed and completed based on various levels of processes; each level of the process is briefly discussed here. In the initial step, the transaction is called by the network node. Once the transaction is received by the network node, then it is sent to other nodes of the network, especially every PC node. Then, by utilizing the SHA256 algorithm, the unique hash value is generated. The newly generated hash values are linked with the previous hash values. Therefore, the transaction with the network is not collapsed. In case of intruders' attempt to append the transaction, the network node validates whether the appropriate candidate is accessing the service based on consensus. Because of this facility, modifying the static ledger is highly impossible. With this process, a secured and reliable system can be enabled with centralized nature. In order to check the genuineness of the user, an effective algorithm is utilized. Once the verification process is done based on the transaction, it is included in the ledger based on the creation of a new block in the network. The essential components of new created block are index, timestamp, preceding hash, current block hash, and data. Following the production of a new block, the most recent block should be used to connect it to the current blockchain. Finally, all the transactions are completed successfully to the network.  Figure 1 shows the complete process.
7. Structure of a block in the blockchain: Figure 2 shows the structure of a block in the blockchain. The first block of the blockchain is known as the genesis block, which does not contain any kind of transaction data. Except for the first block, every block has two fields on its block header, and the second is the body of the block. The body of the block stores all transactions. Block header contains some special type of information such as previous block hash (Merkle root hash of the previous block), difficulty level (shows the difficulty level of consensus algorithm), timestamp (stores time of transaction when it is completed), version (shows the version of used protocol), nonce (this field is used to show PoW), and Merkle root tree (hash of all the verified transactions in the block).
8. Evaluation of blockchain in clinical industry: the clinical data are maintained by the healthcare providers; they generated a massive amount of healthcare data in different forms. These include the medical reports, ledger data, medical imaging, and other measurement data [18]. Therefore, the growth of healthcare data is dramatically increased with a huge database management mechanism. However, still, various issues are existing in the current healthcare system. Therefore, blockchain technology is utilized to deal with these issues that provide security to the healthcare data from being stolen by intruders or attackers [19, 20]. With this technology, authenticating the appropriate user process is executed; therefore, the integrity and efficiency of the data are managed. Moreover, the blockchain system is not needed for multiple levels of verification processes. Here, the data are processed to be visible to every user in the system. Hence, the system can enable the solution to handle various kinds of security challenges in the healthcare domain.

Combining blockchain technology and AI has led to a new era in AI. Many stable applications have been created that allow many users to interact with each other. In this paper, the author uses edge AI to use the power of artificial intelligence (AI). Edge AI is discussed in the next section.

Edge AI: edge AI refers to the dispensation of artificial intelligence procedures at the edge, that is, on devices at the user end. The idea originates from edge computing, which starts from a similar ground: data are kept, handled, and managed right at the IoT (Internet of Things) terminals. Edge AI is not required to connect to the device since the data are treated straight there for machine learning.

Edge AI uses the hardware of the device to process data and for other procedures associated with deep learning and machine learning. How does it work in exercise? Virtual assistants such as Google or Alexa are a decent example. They can learn from end-user phrases or words and save them. IoT devices can respond much faster than traditional Internet connections and do not require the user to be online to perform certain functions. Edge AI is a technology that can provide many benefits to the industry which increasingly trusts IoT devices. We will then list some of these benefits:

1. Improved user experience through reduced latency
2. Integration of wearable technologies such as bracelets and smartwatches
3. Reduced bandwidth requirements and subsequently lower Internet service costs
4. Data processing locally provides greater security and privacy

Figure 3 shows the AI on edge architecture for healthcare. Combining blockchain technology and AI can add worth to healthcare, and biomedical research has a progressive sector. In this paper, the author proposes a novel, distributed approach to measure the worth of time and worth of personal health records in an edge AI-enabled healthcare data sharing on the IBM blockchain platform. This paper provides an overview of AI and blockchain technologies. It can be used to help us accelerate biomedical analysis and advance predictive analysis. Patients are empowered with new tools and techniques to manage their health records. The system helps them to monetize their data by giving them control of their special personal data, and as an incentive benefit, their health is monitored continuously. A blockchain and edge AI approach is extremely streamlined data collection.

The following contributions are made by this study to make personal health record secure, transparent access control, and to develop confidence among diverse stakeholders by using blockchain technology:

1. This paper describes the structure and functionality of a blockchain-based architecture for managing personal health records among a variety of stakeholders. In addition, it highlights how doctors and other medical investigators may gather and access clinical data in a safe, distributed way.
2. A smart contract is built to automate access control procedures to authorized stakeholders.
3. A proof of concept is created using Hyperledger Fabric on IBM platform to illustrate the usability and efficacy of the proposed solution, and a formalised business case is developed. This implementation is intended to facilitate the coordination of different stakeholders of health-related services across several users.

The rest of the paper is organized as follows. Section 2 mainly focuses on literature work based on various techniques, authors, domains, and years. Then, Section 3 focuses on the proposed methodology where detailed information about current techniques, especially blockchain technology in the healthcare industry, is highly discussed. Section 5 focuses on experimental analysis, which provides information about the results obtained by utilizing different performance matrices. The final section describes the conclusion of the entire work.

## 2. Related Work and Motivation

Shahnaz et al. [21] has introduced blockchain technology in the medical field for EHR. The purpose of their system was to make EHR blockchain technology more relevant and accessible to consumers. The proposed structure secures the capability of electronic recordings by categorizing the granular access rules. Besides, this system similarly explores the scaling problem that can be seen by blockchain technology. It was done by using the off-chain stock of records. This system provided the advantages of having a versatile, secure, and necessary blockchain-based solution for EHR architecture. Daraghmi et al. [22], in their paper, created a blockchain-based system called MedChain to oversee medical data. MedChain aims to improve existing systems by providing operational, safe, and successful access to health records by patients, healthcare providers, and other foreigners who care for patients' security. MedChain used time-based smart contracts to oversee transactions and control electronic medical data. This embraced progressed encryption methods for giving further security. This work proposed another motivator instrument that used the level of well-being suppliers concerned their endeavors on keeping up medical records and making new squares. Houtan et al. [23] investigated the block chain (BC)-based self-sovereignty and explored the cutting-edge inpatient data records in the health sector. The goal of the author is to look at the possibilities of BC technology for patient data and identity management. Their inspiration is to explore the potential of technology. As a distribution decentralized technology, BC can be exceptionally valuable, thus empowering patients with their data and self-sovereignty. The focus was on arrangements that focused on acknowledging the underlying electronic health records (EHR) and patient health records (PHR). EHR and PHR are used to record patient data, for example, as noted by a visitor and radiologist. In [24], Akkaoui et al. developed a secure and efficient information management structure which was named EdgeMediChain for sharing health information. The proposed architecture uses both advanced computing and blockchain to ease and enforce healthcare ecosystem requirements for adaptability, security, and protection [25]. Ethereum-based benchmarks showed EdgeMediChain execution efficiency with a nearly 84.75% reduction over 2000 concurrent exchanges. It showed superior performance over conventional blockchain and scalable ledger storage with a linear growth rate. Sui et al. projected an attribute-based branding and attribute renouncement to secure the protection of the client's personality in HSBC in [26]. To safeguard the privacy of the user's identity in HS-BC (Blockchain-Based Healthcare System), an attribute-based signature technique is presented with attribute revocation. The attribute signing key is calculated by combining the attribute master-key and the attribute update-key, where the attribute master-key is related to the user identity and attribute set and the attribute update-key is related to the attribute revocation, under the premise of using attributes to identify users and protect their identities. Through creation utilization of the KUNodes, calculation and attribute disavowal could be adequately accomplished. The planned attribute-based signature scheme required moderately hardly any blending activities and did not depend on a focal power. In [27], Jaiman et al. proposed an implementation of a blockchain-based consent model for data exchange to allow access to selected health information. They used smart agreements to dynamically obtain individual consent for health data and allow data seekers to view and access that information. The dynamic correspondence model resulted in two ontologies: DUO data usage ontology, which models the consent of individual users, and the Access and Automatic Recognition Matrix (ADA-M), which represents questions of users' data requesters. They sent the model to the Ethereum blockchain and evaluated different information exchange situations. This article included the creation of an individual consent model for health data exchange platforms. This model ensures that separate consent is taken into account and that all platform participants are responsible for the exchange of information. In [28], authors proposed a literature review of the proposed block paths for EHR systems. As part of the review, they understood basic information about EHR systems and blockchain before possibly exploring (using) the blockchain in EHR systems. There were also differences found in the difficulties and open spaces. Sharma et al. implemented an EHR upgrade framework using blockchain innovations in [29], and the EHR was kept secure and confidential. Blockchain innovation has retained power over data access through its cryptographic techniques and decentralization. Harmony between information security and openness of information has also been maintained. The main objective of his work was to limit privacy and security concerns in the field of electronic health.

Although various techniques are utilized for effective healthcare management processes, it still requires improving the performance and capabilities of blockchain technology in the healthcare domain. Therefore, the need for enhancing blockchain-based healthcare is highly focused (Table 1).

From the above table, various technologies utilized for blockchain technology are discussed based on different research papers.

### 2.1. Issues Faced on Blockchain Technology

1. Scalability and storage capacity: the capacity of information on the blockchain causes two fundamental issues, i.e., secrecy and scalability. The information on the blockchain is obvious to everybody that is available on the chain; this makes the data disclosure to the all the authorized user, which is not the ideal for healthcare blockchain. which is not the ideal result for a decentralized stage. The information put away on the blockchain would contain persistent clinical history, records, lab results, X-beams reports, MRI results, and numerous different reports; the entirety of this voluminous information is to be put away on the blockchain that would exceptionally influence the capacity limit of the blockchain [16, 23].
2. Lack of social skills: the way blockchain technology works is reasonable by not many individuals. This technology is still in its underlying stages and is continually advancing. Besides, the move from trusted EHR systems to blockchain technology would require some serious energy as clinics or some other medical care foundations need to move their systems to blockchain [20, 25].
3. Lack of universally defined standards: as this innovation is still in the underlying stages and is continually developing, there is no characterized norm for it. Because of this, the execution of this innovation in the medical care division would likewise take additional time and exertion. It would require confirmed guidelines from international authorities that disregard the normalization cycle of any innovation [6]. These widespread guidelines would profit in choosing the information size, information organization, and kind of information that could be put away on the blockchain [37]. Besides, the transformation of this innovation would get simpler because of the characterized principles, as they could be effortlessly implemented in the associations.

## 3. Proposed Methodology

Blockchain is a revolutionary technology that has the potential to help expedite patient data management operations by enabling unparalleled computational efficiency and enforcing trust in a secure manner. In addition, it incorporates a number of notable and built-in features such as decentralized storage and transparency. These characteristics as well as data access flexibility and connectivity enable the broad use of blockchain technology in healthcare data management applications. The blockchain-enabled health systems are shown in Figure 4.

Blockchain relies on the notion of smart contracts to offer terms and conditions that are agreed upon by all of the healthcare partners active in the network, eliminating the need for a third party to function as an intermediary. It lowers administrative expenditures that are not essential. The blockchain is primarily based on three concepts: public key cryptography, peer-to-peer networks, and consensus processes, to name just a few. Blockchains are classified into three groups based on how they manage permission: public blockchains, private blockchains, and consortium blockchains. When it comes to public blockchains, everybody who is connected to the Internet has the ability to join in the consensus mechanism. Rewards and encryption digit verification are included in public blockchains, which are secured by proof-of-work or proof-of-stake methods. The whole public blockchain system is visible, and the identities of any person who participates in it are kept pseudoanonymous by the system. When it comes to private blockchains, only a single entity has complete control over the network's operations. As a result, in order to obtain agreement on such a form of blockchain, a trustworthy agent is required. The consortium blockchain combines the benefits of both public and private blockchain networks in a single system. Specifically, it is only appropriate for particular firms that want to simplify their internal communications with one another. Healthcare businesses may adopt any sort of blockchain network, depending on their individual needs or use case scenarios. Each type of blockchain network has its own set of advantages and disadvantages.

Figure 5 shows the proposed architecture and data flow of system. Because of the dynamic and expanding nature of health data, duplicating all health information to every member of the network would be bandwidth heavy, waste network resources, and create data flow issues. To reap the advantages of blockchain in healthcare, the blockchain would need to serve as an access-control manager for health records and data. An index, or a list of all the user's health records and data, would be included in our proposed health blockchain. The index is akin to a library's card catalogue. The card catalogue includes information on the book as well as a place where it may be located. In the same manner, the health blockchain would function. A user's unique identification, an encrypted link to the health record, and a timestamp for when the transaction was generated would be included in the blocks' transactions. The transaction would include the kind of data contained in the health record, as well as any additional information that would enable commonly used queries, to increase data access efficiency (the metadata could be added as tags). The health blockchain would keep track of an individual user's medical data throughout his life, including official medical records as well as health data through mobile apps and wearable sensors.

All medical data would be housed in a data lake, which would be separate from the blockchain. Data lakes are scalable and can hold a broad range of data, including photos, documents, and key-value stores. Data lakes would be useful tools for health research, and they may be used for a number of analyses, such as looking for characteristics that affect outcomes, selecting the best treatment choices based on genetic markers, and discovering factors that influence preventive medicine. Interactive searches, text mining, text analytics, and machine learning are all supported by data lakes. To maintain data privacy and authenticity, all data stored in the data lake would be encrypted and digitally signed. A digital signature is established when a healthcare professional prepares a health record (prescription, lab test, pathology report, and MRI) to validate its legitimacy. The health data would be encrypted and stored in a data lake. When data are stored to the data lake, a link to the user's health record is added on the blockchain. His health data have been uploaded to his blockchain. Similarly, patients may add digital signatures and encryption to health data via mobile apps and wearable sensors.

The user would have complete control over his data and how it was shared. The user would select who may query and publish data to his blockchain. A mobile dashboard app would show who has access to the user's blockchain. The user may also see who accessed their blockchain and when and what data were viewed. The same dashboard would let the user grant or cancel access to anybody with a unique identity.

Permissions for access control would be more flexible than “all or nothing.” The user would define who has access, the time period for access, and the data categories that may be accessed. The user may change permissions at any moment. On a blockchain, only the user may modify access control restrictions. This creates a transparent environment where the user decides what data are gathered and how they are shared. After gaining access to a user's health data, a provider searches the blockchain for it and uses the digital signature to verify it. The healthcare provider might examine the data using a bespoke best-of-breed application.

To secure the healthcare information, an effective authentication process is required to prevent unauthorized access; this should be executed in every block. Moreover, an effective healthcare system can be achieved by utilizing blockchain techniques. The detailed information about the proposed technological architecture is given below (Figure 6).

The proposed work mainly deals with hospital management issues based on blockchain technology. The given code pattern clearly shows the medical data and the access management platform that has been built using blockchain. Thus, 4 points of view have been given in the platform of applications.

The four layers are as mentioned:

1. *Layer 1*. Solution admin (blockchain operator): the first layer is about the solution admin. This administrator of the solution is the realm of the group of hospitals, and he is one of the hierarchies, who have the highest level of power to access the whole group of management. Therefore, hospitals have the power to join a new organization and appoint hospital administrators who will come under his or her monitoring dashboards. The overall empowerment goes to this solution admin.
2. *Layer 2*. Organization hospital as an admin: the role play of the organization admin is to take care of a particular hospital, which is one of the parts among the group of hospitals. This admin has the potential to join or to make in charge of the new employees either as a doctor or remove the users under his control. The total in charge of a particular hospital goes under this organization admin.
3. *Layer 3*. Doctor pharmacy lab as user: here, in the third layer, the doctor is considered as a user in the company who has a relevant key role and can upload the data of their patients, and also, he can download or can view the data, granted permission to view or download it to their patient records. He is considered as the key person of his patients.
4. *Layer 4*. Patient as a user: finally, the patient is viewed with the appropriate role as a user in the organization and can upload data, view documents of their records for themselves, view document access records, manage access to their documents, and manage the data of their records on their dashboard.

## 4. Implementation and Method

To execute this process, the proposed technique has utilized the Vue.js web app which is incorporated with multiple dashboards within a single page application. With this application, effective real-time communication between the sender and the receiver is done. Then, in the second step, the Node.js server is utilized, which is deployed to Kubernetes container on the IBM cloud platform where the Redis database is incorporated with IBM cloud. With the help of the Node.js server, the effective data storing and retrieving of the data management process can be done by utilizing the Redis database. Then, a REST call is created for an external service. The last step in this process is to use JWT (JSON Web Token) for effective user management.

### 4.1. Ways to Log In

1. The first step in starting a user flow is to log in to their respective dashboards with all partners of applications such as solution manager, hospital administrator, physician administrator, and patient administrator. Solution admin should log in to his respective dashboard by logging in to initiate user flow and then by the other admins.
2. The second step is to log in to the respective dashboards and take them to the login portal of their blockchain solution hosted in the IBM cloud.
3. Finally, the third step is the login portal utilizes the open API link, and then when the user gets login to his dashboard, it generates an on-boarded ID through an identity provider such as IBMID or Google ID. By this, the login process is done successfully which leads to JWT credentials for the user.

### 4.2. Admin Dashboard Process

1. The solution flow management part starts at the management level and, therefore, requires the user to get used to authenticate the login ways listed above.
2. Then, after the successful authentication, the solution admin dashboard can be accessed by the user. Subsequently, by utilizing the admin APIs, the users can be able to access their domain.
3. To process all inquiries from users who have been admin API blockchain solution manager with REST.
4. The ledger updates have been done by the blockchain solution manager that connects with the IBM blockchain platform.

### 4.3. Organization Progress Dashboard

1. Here, the hospital admin flow starts at the organization component, and then the users are required to authenticate themselves by the login ways as described above.
2. Next to their successful authentication, the hospital admin dashboard can be accessed by the users. With this, they can add or remove any user in their corresponding hospital-like as the doctor or the patient with the on-boarded rules by using the organization APIs in our case.
3. Through REST, the blockchain solution manager has been connected with all the organization APIs to the process the queries of the users.
4. Ledger update process integrated with 0020 blockchain solution manager into the IBM blockchain operating system.

### 4.4. Steps of Doctor Dashboard

1. The physician flow begins with the physician components, and then here users must authenticate themselves in the login ways as mentioned above.
2. Then, after their successful authentication, the doctor dashboard can be accessed by the users. In this case, they can view the patient's medical record as part of the hospital, and they can download any medical records of the patient and have access to view it using the medical API.
3. The status of the use of ACL for all patient's documentation is maintained by the ACL document as explained below.
4. Blockchain document store through REST: it has been connected with all the doctor APIs to process queries of the users.
5. The updated ledger is integrated with the IBM blockchain operating system by blockchain document store.

### 4.5. Patient Domain

Thus, the components of the patient begin to flow, and then the users must authenticate themselves using the above-given login.

Then, for their successful authentication, the user can access the patient's dashboard and they can upload medical data for themselves, download any of their medical data, view the access logs of their documents, and view their documentation using the patient's API. The application level of the ACL for all documents was maintained by the ACL flow as described below. All patients are connected to the blockchain document store via AAPI's REST to process user queries. Blockchain document store is integrated with the IBM blockchain operating system and updates the ledger properly.

### 4.6. The Flow of the Document Access Control List (ACL)

1. To manage the document level access control across hospitals, the physician, patient components, and Redis APIs are linked, which uses techniques of management.
2. The Redis API speaks to a Node.js server parked in the doctor container in the Kubernetes cluster in the IBM cloud.
3. The two servers in the databases and that entries to the document should be or have been granted on behalf of each user.

## 5. Experimental Results and Discussion

In this segment, implementation outcomes of the developed technique are verified. The experimental results in this section demonstrate the effectiveness and achievability of the proposed method. We have evaluated our work with various performance matrices to examine the presentation and effectiveness of the propounded strategy. We divided the experiment results into two categories: one is Scenario 1 for basic experiment results such as Recall and Confusion metrics, and Scenario 2 is benchmark performance analysis results such as latency, throughput, and commit time. Of the proposed system, both scenarios are performed under predefined simulation settings for hardware and software as discussed in the next section.

### 5.1. Simulation Settings

Table 2 shows the simulation setting for hardware and software. We use IBM cloud private to test our proposed system. Hyperledger fabric is used to implement the proposed system; for this, we used IBM Blockchain Platform 2.0 as a service on IBM cloud. Our fabric network has 2 organizations and 2 peers, each with one ordering service with 2 CA. our network uses CouchDb to store peer data. To analyze the performance of our network, we use Hyperledger Caliper. Further configuration settings are shown in Table 2.

Resource allocation is very important when we install IBM blockchain on ICP (IBM Cloud Private) platform. Each element (Orderer, Peer, and CA (certificate authority)) of the Hyperledger Fabric platform requires memory (RAM), a virtual core processor (vCPU), and storage to store data. Each element needs some resource allocation, depending upon the design of the blockchain network. During this experiment, we use the default configuration for resource allocation, as shown in Table 3.

### 5.2. Scenario 1: Basic Experiment

Several remarks are taken into the justification for evaluating and understanding the proposed system. We have evaluated our work with various performance matrices to examine the presentation and effectiveness of the propounded strategy. Some of them are explained below.

*Evaluation matrices* are shown in Table 4.

Detection rate (DR) and false positive (FP) are used to estimate the performance of the intrusion detection system, which are given in the following equations:

(1) $$\begin{array}{c} \mathrm{DR}=\frac{\mathrm{total}\;\mathrm{detected}\;\mathrm{attacks}}{\mathrm{total}\;\mathrm{attacks}}\mathrm{\times 100},\\ \mathrm{FP}=\frac{\mathrm{total}\;\mathrm{misclassified}\;\mathrm{process}}{\mathrm{total}\;\mathrm{normal}\;\mathrm{process}}\mathrm{\times 100,}\\ \mathrm{Accuracy}=\frac{\mathrm{TP+TN}}{\mathrm{TP+TN+FP+FN}},\\ \mathrm{Detection}\;\mathrm{Rate}=\frac{\mathrm{TP}}{\mathrm{TP+FP}},\\ \mathrm{False}\;\mathrm{Alarm}=\frac{\mathrm{FP}}{\mathrm{FP+TN}}, \end{array}$$

where FN denotes false negative, TN denotes true negative, TP denotes true positive, and FP denotes false positive.

Recall:

(2) $$\begin{array}{c} \begin{array}{c} \mathrm{Recall=}\frac{\mathrm{TP}}{\mathrm{TP+FN}} \end{array}. \end{array}$$

Precision:

(3) $$\begin{array}{c} \begin{array}{c} \mathrm{Precision=}\frac{\mathrm{TP}}{\mathrm{TP+FP}} \end{array}. \end{array}$$

F1 Score:

(4) $$\begin{array}{c} \begin{array}{c} F1\;\mathrm{Score=2*}\left(\mathrm{Precision*Recall}\right) \end{array}. \end{array}$$

Area under ROC curve: the essential term in area under ROC curve is TP/Recall/Sensitivity:

(5) $$\begin{array}{c} \mathrm{TP}/\mathrm{Recall}/\mathrm{Sensitivity}=\frac{\mathrm{TP}}{\mathrm{TP+FN}},\\ \mathrm{Specificity}=\frac{\mathrm{TN}}{\mathrm{TN+FP}},\\ \mathrm{FP}=\frac{\mathrm{FP}}{\mathrm{TN+FP}}. \end{array}$$

The results of our proposed system are given by graphical representation in the following section.

Figure 7 shows the results obtained from the Recall measure calculation processes. With these results, the proposed methodology produced much better results than the existing techniques.

Figure 8 shows the results obtained from the F1 Score calculation processes. In this graph, the dot represents F1 Score, and the cross line represents the ROC curve.

Figure 9 illustrates the graphical results of the proposed work by analyzing the prediction of fraudulent and nonfraudulent activities. For this calculation, a confusion matrix calculation is performed to produce these results. Also, confusion matrices mainly fall into two classes: true class and predicted class. Thus, the proposed methodology is more effective than the existing ones.

### 5.3. Scenario 2: Benchmark Performance Analysis

Several observations are taken into consideration for evaluating and understanding the proposed system. The first test is conducted with different parameters and is performed in three rounds of reading/writing the data into the ledger. Every round has 1000 transactions with different transaction rates. The transaction arrival rate is varied from 50 to 250 transactions per second. We choose three scenarios of the network to measure the performance, one is 2org2peer, the second is 2org1peer, and the third is 1org1peer.

Figure 10(a) shows the transaction commit time; it gives the performance of the network according to the time taken to complete a transaction. Time from 20 seconds to 140 seconds with 20-second intervals is shown on *x*-axis. The number of transactions from 1000 to 4000 with an interval of 1000 is shown on *y*-axis. All three scenarios, 2org2peer, 2org1peer, and 1org1peer, portray different behaviors of the transactions. The results are collected in three different rounds with different transaction rates. The 2org2peer is consuming 140 seconds of the network to reach 2300 transactions. On the other hand, at the same time, 2org1peer completes 2700 transactions and 1org1peer completes 3100 transactions. It is clear from the results that, with the increase in the number of organizations and peers in the network, the time required to complete transactions is also increasing.

The graph in Figure 10(b) shows the average latency with respect to transaction rate for different organizations having different numbers of peers. Average latency measured in time is shown on *y*-axis from 0 seconds to 60 seconds with a 10-second interval. Transaction rate is in TPS (transaction per second) shown on the *x*-axis from 50 to 250 with an interval of 50. The graph shows that the latency in the case of 2org2peer is very high as compared to 2org1peer and 1org1peer at the transaction rate of 50 TPS. At 250 TPS, 2org2peer has 33.12 latency, whereas 2org1peer and 1org1peer have 23.12 seconds and 11.34 seconds latency, respectively. The minimum latency of 3.13 seconds is achieved for 1org1peer at 50 TPS. The highest latency 33.12 is for 2org2peer at a transaction rate of 250 TPS. The graph concludes that when we increase the transaction rate from 50 TPS to 250 TPS, latency increases in all three cases.

The graph in Figure 10(c) shows the throughput with respect to transaction rate for the different organizations that have different numbers of peers. Throughput measured in the number of successful transactions per second is shown on *y*-axis from 0 to 150 with 25 intervals. Transaction rate is in TPS (transaction per second) shown on the *x*-axis from 50 to 250 with an interval of 50. The graph shows that the throughput is approximately the same in all cases at 50 transaction rates. The throughput reaches the highest 124 TPS for 1org1peer, while 2org2pper and 2org1peer decrease the throughput to 114 and 119, respectively, at 250 transaction rates. The graph concludes that when we increase the transaction rate from 50 to 150, throughput increases in all three cases and have the approximately same value, but after 150 to 250 transaction rates, throughput gets saturation point in all the cases; hence, throughput values do not increase like before.

The querying latency is analyzed for three cases, 2org2peer, 2org1peer, and 1org1peer, working at different transaction rates, as shown in Figure 11(a). Transaction rate is measured in transactions per second and is depicted on the *x*-axis ranging from 50 to 250. Latency is depicted on the *y*-axis ranging from 5 to 30. This graph gives two major observations: one is for variation in latency for different transaction rates and the other is for the impact of the different number of organizations and peers on latency. The latency usually increases with the increase in transaction rate; as for the 1org1peer, the latency became almost 5-folds from 50 TPS to 250 TPS. The dependency of organization and peers on latency also depicts that with the increase in the number of organizations and number of peers, the latency also increases. The increase in latency with organization and peers is a minimum of 3-fold in almost all TPS. Therefore, the conclusion from this graph is that minimum latency is achieved for 1org1peer at a transaction rate of 50 TPS and maximum is for 2org2peer at a transaction rate of 250 TPS.

To analyze querying throughput for the different number of organizations and peers, different transaction rates are used, as shown in Figure 11(b). The transaction rate taken in transaction per second is shown on the *x*-axis ranging from 50 TPS to 250 TPS. Throughput is on the *y*-axis ranging from 25 to 150. The first observation from this graph is that throughput is rapidly increasing with the increase in transaction rate from 50 TPS to 150 TPS, but after that, the graph becomes linear. This shows that after a saturation point, the throughput does not increase. The second observation is for the different number of organizations and peers, that is, throughput at any transaction rate value is highest for 1org1peer and lowest for 2org2peer. At 50 transaction rates for all 3 cases, throughput are almost 50 but at 250 TPS, it is not more than 124.

Figure 12 shows how latency is varied according to block size. The latency is analyzed for two cases, block size 5 and block size 10, working at different transaction rates, as shown in the graph. Transaction rate is measured in transactions per second and is depicted on the *x*-axis ranging from 50 to 250. Latency is depicted on the *y*-axis ranging from 0 to 70. It is clear from the graph that latency is more in block size 10 as compared to block size 5 at 50 transaction rates, but when we increase the transaction rate from 50 to 250, latency is high for block size 5 as compared to block size 10.

Several studies and applications addressing the use of blockchain to solve security concerns in healthcare systems have recently been published. We discuss some of these studies in this part, and Table 5 summarizes their authors, publication year, and technique implementation. The table also shows the primary obstacles addressed in each study, as well as the main distinctions between them in terms of blockchain type and whether or not the work considered data encryption, scalability, and interoperability concerns.

## 6. Security Analysis

The development of blockchain technology is still in progress and not in final stage. It is not only the technology that is at risk, but also the application itself. When it comes to blockchain security, the majority of researchers now focus on three primary areas: integrity, privacy, and scalability. In this paper, the author also focuses on the same issues along with data transmission.

A smart contract's access control rules or a network-level channel may be used to ensure data privacy. As a result, only those who have the proper credentials may access the ledger, limiting the amount of information that can be accessed. It is necessary for the transaction peer to be recognized by the channel before it may join the channel and participate in transactions. Declarative access control is provided by the network's access control rules. Setting access control rules allows us to specify which network users may execute a specified action on a given object.

The integrity of the blockchain is safeguarded by the presence of proof of work and the enormous number of honest miners. Even while the blockchain offers anonymity, it cannot be relied upon to protect your personal information. The attacker may, however, use incoming and outgoing traffic and transaction data to conduct some mapping. In order to secure your privacy on the blockchain, you have two options right now: one way is to use a technology like “safe transmission” to provide an anonymous protective measure to an existing blockchain. Other options include creating a whole other chain of ledgers, such as Zerocash, which uses new primitives in its block to ensure complete anonymity. The foundation of blockchain technology is based on cryptography. Until the hash function or encryption technique is safe, the blockchain's security cannot be guaranteed. There is no doubt that the SHA256 hash function and elliptic curve cryptography employed in the blockchain are secure, but emerging technologies such as quantum computing have raised concerns about their long-term viability. As a consequence, we must keep abreast of recent developments in the field of algorithm security and work to develop new ones.

Even if blockchain technology is now plagued by a number of security issues, each new technology must go through a process of continual problem fixing in order to mature. Blockchain qualities such as tamper resistance and decentralization may be used to address issues in various sectors.

## 7. Discussion

Are there any issues which need to be focused that have not yet been addressed? Incorporating blockchains into current healthcare infrastructures is not without its challenges. The first consideration is system scalability. While the data saved on the chain may be managed, the number of patients and parties participating will expand with time. Computing resources, such as processing power and storage capacity, are finite. This may impede blockchain services. This may become an issue due to the network's continued development, scalability, and resource requirements. Another concern is the idea of “garbage in, garbage out” (GIGO). This is a case when a user enters inaccurate or random data. To handle this data, the system may produce mistakes or erroneous results. Healthcare blockchains may encounter the same problem. Now that the patient is involved in their own treatment, “garbage” may be entered. A caretaker or other professional with modification or writing authorization may face the same risk. Malicious users who want to exploit security flaws to steal data or inflict damage will always exist. Even if the blockchain is safe, end-point security is still a concern. An attacker may pollute the blockchain if an end user is hacked. They may take data from the hacked victim and supply bogus information to be submitted in the chain.

Can blockchains be used in conjunction with artificial intelligence to improve the quality of personalized healthcare even more? Data science is also trying to enhance healthcare by using AI and machine learning techniques. Like blockchains, these judgments are decided by algorithms. While blockchains gather data to guarantee data integrity, AI strives to forecast and make intelligent judgments. Examples of healthcare choices include medical diagnosis, drugs, and treatments. Blockchain systems have improved data integrity and prevented conventional threats. Large volumes of data cannot be sent directly via the blockchain without affecting system speed and data security. By incorporating AI algorithms into the system, data may be processed in advance, leaving just results and information on the blockchain. A healthcare practitioner can still understand how data were handled and why intelligent judgments were made since the blockchain audits all transactions. To make correct conclusions, the data used must be dependable. Given the immutability and trustworthiness of blockchain data, the dataset acquired by machine learning algorithms would allow for appropriate decision-making. Data scientists no longer need to manually process data needed by AI systems. The capacity of AI to make intelligent judgments may also help with block mining, decreasing the need for processing resources. Using machine learning algorithms to mine blocks instead of conventional ways may save time and money. If a healthcare professional has appropriate authorization to access trustworthy patient data, then AI may be used to categorize patients based on molecular profiling, chemical response, gene variants, hereditary illness, or any other profile.

## 8. Limitation of the Proposed System

This section outlines the constraints of the proposed work. One thing to note is that although it is practically difficult to hack and tamper with information kept in the blockchain, this is not true of the programming instructions included inside the smart contract. A simple programming error might set off a cascade of events that would be catastrophic. This is a situation that merits our attention and needs our undivided attention. Another drawback of the blockchain network is connected to the consensus mechanism that is utilized to achieve consensus. The Practical Byzantine Fault Tolerance (PBFT) mechanism, which is utilized in the proposed blockchain platform, may be deactivated if more than a third of the peers are offline at the same time [32]. The occurrence of this incidence is possible in small networks with a restricted number of peers. The number of peers must be increased in order to prevent hostile peers from taking over the whole system.

## 9. SWOT Analysis

SWOT (Strengths, Weaknesses, Opportunities, and Threats) analysis is a practice for evaluating the abovementioned IV facets of the proposed architecture.  Figure 13 shows the complete SWOT analysis of the proposed healthcare system using blockchain.

## 10. Conclusion

In this technological world, the utilization of blockchain technology is ubiquitous, which is an active research topic in recent days. Therefore, many research works are incorporated into this area to enhance their performance and ability. Our proposed work is highly based on blockchain technology in the field of healthcare processing. Therefore, we analyze the current techniques and the existing problems of the healthcare domain. In this paper, we focus on blockchain for an effective healthcare management process. Combining blockchain technology and AI can add worth to the healthcare and biomedical research sector. In this paper, the author proposes a novel, distributed approach to measure the worth of time and worth of personal health records data sharing on the IBM blockchain platform. With the utilization of our work, the problem in the blockchain-based healthcare management system is reduced, especially the traditional blockchain system usually decreases the latency. Therefore, the proposed technique is highly focused on improving latency. The result of our proposed system is calculated based on various matrices, such as F1 Score, Recall, and Confusion matrices. Therefore, the proposed work scored high accuracy and better result.

Current healthcare systems must address the lingering security and privacy concerns that patients have in order for them to have more trust in their medical professionals and the clinics where they get treatment. The administration of electronic medical records (EMRs) is a critical topic that requires attention. The digitization of medical records has made it easier to store and distribute them. The challenges of illegal access and disclosure, the centralized system that may be seen as a single point of attack, and patient medical information segmentation in the event that numerous healthcare practitioners are visited continue to be a concern. As a means of addressing these problems, academics are turning to blockchains, a technology that was initially presented with the introduction of Bitcoin. Over time, various improvements have been made to the initial blockchain architecture, allowing it to be utilized for a variety of purposes more than simply cryptocurrencies and financial transactions. Researchers have started investigating the potential applications of blockchain technology in order to enhance the present healthcare system. Blockchains may be utilized as a digital ledger to facilitate communication between patients, caregivers, and insurance companies because of their irreversible, transparent, distributed, and decentralized nature. It is also possible to consolidate patient information into a single file, making it more thorough and providing caregivers with a better perspective of the patient's health history.

The integration of blockchains into healthcare infrastructures has a lot of promise, as has been shown. This field will continue to benefit from research, which will be advantageous to healthcare professionals, patients, and other parties engaged in it, such as research institutes and insurance companies. Once the remaining concerns with blockchains are resolved, healthcare systems will be able to adapt to the advantage of all stakeholders.

## Figures and Tables

**Figure 1:** Blockchain transaction process.

**Figure 2:** Structure of a block.

**Figure 3:** AI on edge architecture for healthcare.

**Figure 4:** Blockchain-enabled healthcare systems.

**Figure 5:** Proposed architecture (credit: http://www.healthit.gov; Frost & Sullivan).

**Figure 6:** The technological architecture.

**Figure 7:** The graph showing the Recall measure.

**Figure 8:** The graphical representation of F1 Score (dot) for ROC (line).

**Figure 9:** The confusion matrices.

**Figure 10:** (a) Transaction commit time, (b) transaction average latency, and (c) transaction throughput.

**Figure 11:** (a) Querying time transaction latencies. (b) Querying time transaction throughput.

**Figure 12:** Transaction latency with varying block size.

**Figure 13:** SWOT analysis.

**Table 1:** Blockchain-based issues and techniques.

Author	Ref.	Issues focused	Contribution	Year
Ayesha Shahnaz et al.	[21]	Scalability, storage, and capacity	Off-chain storage mechanism of IPFS	2019
Eman-Yasser Daraghmi et al.	[22]	Large dataset at low latency	MedChain with ElGamal re-encryption	2019
Bahar Houtan et al.	[23]	BC-based EHR and PHR are essential to realizing a distributed autonomous healthcare ecosystem	IoT, research and trial, supply chain, and healthcare insurance	2020
Raifa Akkaoui et al.	[24]	Interoperable, secure, and successful access	BC-based EHR and PHR	2020
Qianqian Su et.al.	[26]	To safeguard the privacy of the user's identity in HSBC	KUNodes algorithm for attribute renovation in the healthcare system	2020
Vikas Jaiman et al.	[27]	To automate a generic consent model, and the solution is deployed and tested in LUCE	The Data Use Ontology (DUO) and the Automatable Discovery and Access Matrix (ADA-M)	2020
Shuyun shia et al.	[28]	Operational challenges	A fully integrated blockchain technology with existing EHR systems	2020
Yogesh Sharma et al.	[29]	Security, decentralization, and transparency	Cryptography based on hashing	2020
Faisal Jamil et al.	[30]	Drug supply chain integrity	Untimely access to electronic medication and patient records is granted through smart contract	2019
Lei Hang et al.	[31]	Improve data transparency	A secure blockchain platform for clinical data. The smart contract assures traceability, avoids a posteriori reconstruction, and securely automates clinical trial activities	2021
Lei Hang et al.	[32]	EMR integrity management	The suggested smart contract to secure EMR administration gives patients a full, immutable record and simple access to their medical information across hospital departments	2019
Helen Sharmila et al.	[33]	Wireless body area network (WBAN)-IoT	Proposed the EiA-H2B model (edge intelligent agent hybrid hierarchical blockchain)	2021
Weizhi Meng et al.	[34]	Trust management against insider attacks	Improve the Bayesian inference-based trust management of MSNs by using blockchains to make it more effective	2020
Guipeng Zhang et al.	[35]	Privacy preserving EHR in cloud	Establishing secure payment procedures with the use of blockchain-based smart contracts, which may allow patients and hospitals to pay for diagnostic and storage services in a dependable manner	2022
Wei Yang Chiu et al.	[36]	Secure data sharing and access scheme	Design a scheme that uses smart contract and blockchain to provide a secure data sharing and access environment	2021

**Table 2:** Simulation configuration for hardware and software.

Software configuration	Hardware configuration
IBM Cloud Private 3.1.0	Operating system: Windows 10 64 bit
IBM Blockchain Platform 2.0	System manufacturer: LENOVO
Ubuntu 16 LTS	BIOS : EFCN50WW (type: UEFI)
Hyperledger Fabric 2.1 on IBM cloud	Memory: 8192 MB RAM
IBM cloud worker node is deployed with Hyperledger Fabric consisting of 2 CAs, 2 peers, and 1 orderer	Processor: Intel© core™ i7-10750H CPU @ 2.60 GHz (12 CPUs), ∼2.6 GHz
CouchDB is used to store peer data	Network: 1Gbit/s
Caliper is used for benchmark	HDD/SDD : 1 TB/512 GB
	Gpu : NVIDIA GeForce 1650 4 GB

**Table 3:** Default resource allocations for IBM blockchain platform.

Component (all containers)	vCPU	Storage (GB)	Memory (GB)
CA	0.1	20	0.2
Ordering service	.45	100	0.9
Peer	1.7	200	3.0
Total	2.25	320	4.1

**Table 4:** Parameters and definition.

Parameters	Definition
True positive or detection rate	Unauthorized access occurs and the alarm raised
False positive	No unauthorized access but alarm raised
True negative	No unauthorized access and no alarm
False negative	Unauthorized access occurs but no alarm

**Table 5:** Comparison summary of different proposed blockchain framework in healthcare.

Authors and reference	Application type	Blockchain type	Year	Contribution	A	B	C
Griggs et al. [19]	Securing IoT medical devices	Private	2018	Authors focus to maintain the data integrity and privacy of healthcare data	No	No	Yes
Liang et al. [38]	EMR management	Public	2017	Proposed a method to maintain the privacy and data integrity of healthcare data	Yes	Yes	Yes
Azbeg et al. [39]	Securing IoT medical devices	Private	2018	In this paper, authors developed a method to ensure the data integrity, confidentiality, privacy, and access control for medical data	No	No	Yes
Huang et al. [40]	Drug traceability	Private	2018	The authors proposed a framework to maintain the privacy and authenticity of healthcare data	Yes	No	No
Kumar et al. [41]	Drug traceability	Private	2019	To develop a secure system for traceability and access control	No	No	Yes
Dagher et al. [42]	EMR management	Private	2018	Proposed a method for data integrity, privacy, and access control for EHR data	No	Yes	No
Hathaliya et al. [43]	Remote patient monitoring	Private	2019	The authors proposed a method for integration of decentralized artificial intelligence	No	No	No
Sahoo et al. [44]	Drug traceability	Private	2019	The authors proposed a drug traceability system	No	No	No
Jamil et al. [45]	Remote patient monitoring	Private	2020	The authors work on the data integrity, privacy, and access control for EHR data	Yes	No	Yes
Torky and Hassanien [46]	Tracking COVID-19	Not specified	2020	The authors proposed a framework for data privacy for COVID-19 patient data	No	Yes	No
Xu et al. [47]	Tracking COVID-19	Private	2021	To develop a system for data integrity and traceability for COVID-19 patient data	Yes	No	Yes
The proposed approach	PHR management	Private	2022	Proposed a novel framework for personal health record (PHR) management using IBM cloud data lake and blockchain platform for an effective healthcare management process	Yes	Yes	Yes

A, scalability; B, interoperability; C, data encryption.
